The article "Citrate stabilized Fe3O4/DMG modified carbon paste electrode for determination of octamethylcyclotetrasiloxane in blood plasma and urine samples of cement factory workers" was retracted in 2022. Reasons: unreliable results or conclusions; bias or lack of balance; concerns about the data; concerns about the results or conclusions.

# Citrate stabilized Fe_3_O_4_/DMG modified carbon paste electrode for determination of octamethylcyclotetrasiloxane in blood plasma and urine samples of cement factory workers

**DOI:** 10.1186/s13065-020-00681-7

**Published:** 2020-04-08

**Authors:** Rashid Heidarimoghadam, Abbas Farmany

**Affiliations:** 1 Health Sciences Research Center and Department of Ergonomics, School of Public Health, Hamadan University of Medical Sciences, Hamadan, Iran; 2 Dental Research Center, Hamadan University of Medical Sciences, Hamadan, Iran

**Keywords:** Octamethylcyclotetrasiloxane, Voltammetry, Human fluids

## Abstract

In this paper, a novel mercury-free electrochemical probe was constructed for the trace determination of octamethylcyclotetrasiloxane (D_4_) in some biological fluids by adsorptive stripping voltammetry. The platform is based on the adsorptive accumulation of Ni(II) onto a carbon paste electrode modified with citrate stabilized Fe_3_O_4_ (Cit-Fe_3_O_4_) and dimethylglyoxime (DMG). It was shown that trace levels of D_4_ enhance the electrochemical adsorptive stripping signal of Ni(II) on the electrode platform. It was shown that electrochemical signals are proportional to concentrations of D_4_. The supporting electrolyte, pH and instrumental parameters associated with the electrode response, including scan rate, accumulation potential and deposition time were optimized. The electrode platform demonstrated well resolved, reproducible peaks, with relative standard deviation (RSD) of 3.8% and detection limit (3S_b_/m) of 27.0 ng/mL. The sensor exhibited good D_4_ detection and quantification in human blood plasma and urine samples.

## Introduction

As low molecular weight (LMW) compounds, siloxane derivatives play a vital role in human life. Today, the ever-increasing development of silicon technology has resulted in more than 150,000 products in pharmaceutics, medicine, cosmetics, and food industry [1–3]. It is estimated that global siloxane market reached over 19 billion dollars [3, 4]. Many devices and tools used by infants, adults as well as the elderly are made of siloxane derivatives. Today, 50% of new skin care products contain one of silicon derivatives [3, 5]. Recent studies showed that some of siloxane derivatives may interfere with the function of the endocrine glands and may adversely affect the fertility [5–8]. It was shown that siloxane derivatives such as octamethylcyclotetra-siloxane (D_4_), decamethylcyclopentasiloxane (D_5_) and dodecamethylcyclohexa-siloxane (D_6_) can cause cancer or inflammation in the glands [5–7]. The molecular structure of D_4_ is shown in Scheme 1. Most common siloxane polymer used in medical products is PDMS, which has been widely used in breast implants. It has been reported that silicon migrates from the implant to specific tissues such as plasma and blood [6, 7]. So the monitoring of siloxane derivatives, especially in human body fluids, is important.

**Scheme 1:** Molecular structure of D_4_

Siloxane derivatives may be detected using inductively coupled plasma spectroscopy (ICP), gas chromatography (GC), and high performance liquid chromatography (HPLC) [6–16]. However, some methods can detect the silicon element alone, and detection of organosilicon compounds remain an issue.

Recently, electrochemical methods with excellent selectivity and sensitivity have been developed for trace analysis of micro/macro molecules in biological samples. At this time, carbon based electrodes are modified using different nanomaterials to achieve the best sensitivity. Superparamagnetic iron oxide nanomaterial (Fe_3_O_4_) is a typical solid of layered metal oxides of Fe_2_O_3_ and FeO. In the structure of this metal oxide nanocrystal, one of two tetrahedral interstitial sites is filled by Fe^3+^ cations and other site is occupied by Fe^2+^ and another half of Fe^3+^. In these typical metal ions, valence mixing decreases the resistivity and possesses an excellent conductivity [17]. Also, surface to volume ratio and specific surface area of this nanomaterial accelerates the electron flow and increases its effective contact with electrolyte, which leads to excellent electrosensing ability [18–21].

To the best of our knowledge, at this time no electrochemical method was reported for the quantification of siloxane derivatives in real samples. The aim of this work was to obtain a mercury-free electrode for quantification of octamethylcyclotetrasiloxane (D_4_) in some biological fluid samples using a modified carbon paste electrode (CPE). To enhance the sensitivity, carbon paste electrode was modified with Cit-Fe_3_O_4_ and dimethylglyoxime (DMG) as selective chelating agent. The developed Cit-Fe_3_O_4_-DMG CPE sensor exhibited excellent electrochemical performance and obtained high sensitivity toward D_4_. Meanwhile, the interference of some coexisting ion/molecules was investigated. The reproducibility and stability of the fabricated electrode were also investigated. Moreover, the potential of the sensor was verified by analyzing D_4_ in blood plasma and urine samples.

## Experimental

All experimental protocols were approved by the Ethics and Animal Handling Committee of the Hamadan University of Medical Science (IR.UMSHA.REC.1395.99). All methods were carried out in accordance with relevant guidelines and regulations. Oral consent was obtained from all participants.

### Apparatus

Electrochemical experiments were made using an Autolab potentiostate/galvanostate (Ecochemie, Netherland). A personal computer was used for data storage. A carbon paste electrode was used as working electrode. A platinum wire and a silver/silver chloride electrode were utilized as counter and reference electrode, respectively.

### Materials

Ferric chloride hexahydrate (FeCl_3_·6H_2_O) and nickel chloride hexahydrate (NiCl_2_·6H_2_O) were purchased from Merck (Germany). Octamethylcyclotetrasiloxane (D_4_) was purchased from Sigma (USA). Dimethylglyoxime (DMG) was purchased from Sigma-Aldrich (USA). Stock solution of Ni^2+^ was prepared by dissolving an appropriate amount nickel chloride in double distilled water. Acetate-acetic acid (HAc-NaAc) buffer was used to adjust the pH of solutions. D_4_ solution was prepared by dissolving 25 mg of D_4_ in 25 mg of ethyl acetate and H_2_O (50:50 w/w). Different concentrations of D_4_ were prepared by diluting the stock solution with double distilled water.

### Synthesis of Cit-Fe_3_O_4_

Fe_3_O_4_ nanocrystal was synthesized using an improved solvothermal method [21]. Briefly, 0.32 g FeCl_3_·6H_2_O and 0.1 g trisodium citrate were dissolved in ethylene glycol. 0.6 g sodium acetate was added to the solution and it was homogenized ultrasonically for 1 h at room temperature. The solution was transferred into a chemical autoclave and aged for 10 h at 200 °C. After cooling at room temperature, the nanocrystals were decanted and washed with acetone and pure ethanol. Finally, the synthesized Fe_3_O_4_ was ethanol evaporated using a reduced pressure chamber.

### Sensor preparation

The unmodified carbon paste electrode was prepared by mixing 0.1 g graphite powder and 0.2 mL paraffin oil. A portion of the resulting paste was then firmly inserted into the electrode cavity (2.6 mm diameter). Electrical contact was made through a copper wire. The Cit-Fe_3_O_4_-DMG CPE electrode was prepared by mixing appropriate amounts of graphite powder, Cit-Fe_3_O_4_ nanoparticles, DMG powder and paraffin oil. The surface of modified/unmodified electrode was thoroughly washed before each measurement by double distilled water.

### Procedure

Ni^2+^ and 0.05 mol L^−1^ HAc-NaAc buffer (pH 4.65) were transferred into a three electrode electrochemical cell setup. Cit-Fe_3_O_4_-DMG-CPE was immersed into the cell as working electrode. The electrochemical cell was degassed with nitrogen gas for 2 min. An accumulation potential of – 0.2 V was applied to working electrode. After 100 s stirring, the potential was scanned at rate of 120 mV s^−1^ in differential pulse waveform mode.

## Results and discussion

### Synthesis and characterization of Cit-Fe_3_O_4_

The Cit-Fe_3_O_4_ nanocrystals were solvothermally synthesized and characterized using Fourier-transform infrared spectroscopy (FTIR), X-ray powder diffraction (XRD), vibrating-sample magnetometer (VSM), scanning electron microscope (SEM) and transmission electron microscopy (TEM). FTIR spectra of Cit-Fe_3_O_4_ is shown in Fig. 1a. The characteristic peak at 578 cm^−1^ is related to the vibration of Fe–O bond which confirms the magnetic phase of nanoparticles. Absorption peaks at 1371-1540 cm^−1^ confirms the stretching vibration (symmetric and asymmetric) of carbonyl groups [21].

**Fig. 1:** **a** FT-IR spectra; **b** XRD pattern; **c** Magnetization hysteresis loop of Cit-Fe_3_O_4_

The microstructure of Cit-Fe_3_O_4_ nanocrystal was characterized by the x-ray diffraction (XRD) technique. Figure 1b shows the XRD pattern of magnetic nanocrystals. Indexing 2θ diffraction peaks at 30.0, 35.6, 43.8, 54.2, 57.2 and 62.5 to (220) (311) (400) (511) and (440) shows the cubic spinel structure of nanocrystals. The result of this study is in accordance with the standard PDF card (JSPDS 86-2343) of magnetite. The magnetic characteristic of Cit-Fe_3_O_4_ nanocrystals was evaluated by a vibrating-sample magnetometer (VSM). The nanocrystals exhibit superparamagnetic behavior and have lower saturation magnetization value than the bulk magnetization (~ 92 emu/g) [22]. Magnetization hysteresis loop of Cit-Fe_3_O_4_ is shown in Fig. 1c. VSM data shows a superparamagnetic behavior of synthesized nanocrystals with a saturation magnetization of 50.7 emu/g. The saturation magnetization and susceptibility of Cit-Fe_3_O_4_ seems to be smaller than Fe_3_O_4_. This is due to the existence of citrate diamagnetic shell surrounding the Fe_3_O_4_ which quench the magnetic moment [23]. However, Cit-Fe_3_O_4_ showed superparamagnetic behaviors, which indicate that magnetite nanocrystal is incorporated in the composite particles, which exhibited no residual magnetism effect at applied magnetic field from the hysteresis loops. Surface micromorphology and topography of as-prepared Cit-Fe_3_O_4_ nanocrystals was characterized by scanning electron micrography (SEM). As indicated in Fig. 2a, the irregular shape of nanocrystals with excellent dispersity is observed. TEM image of nanocrystal is shown in Fig. 2b. The size of Cit-Fe_3_O_4_ nanocrystals is estimated as 150 nm. Surface zeta potential of Cit-Fe_3_O_4_ at different pHs was evaluated and the surface charge of nanocrystals was obtained. As shown in Fig. 2c, the zeta potential of Cit-Fe_3_O_4_ at optimum pH of this method (pH 4.65) is – 9.0 mV.

**Fig. 2:** **a** SEM; **b** TEM micrograph; **c** Zeta potential of Cit-Fe_3_O_4_

### Electrochemical experiments

Cit-Fe_3_O_4_-DMG-CPE electrode was prepared and its indirect electrochemical response to D_4_ molecule was studied. Accumulation potential applied onto the electrochemical cell pre-concentrates the nickel ion on the working electrode surface in an open circuit conditions. The possible mechanism for enhanced stripping signal of D_4_ could be related to high electron density on the D_4_ molecule surface which follows the reversible redox process of Ni^2+^/Ni^0^ pair. Nickel redox peak is registered at -0.91 V at Cit-Fe_3_O_4_-DMG-CPE electrode surface. In the presence of nickel ion, introducing trace levels of D_4_ onto the electrochemical cell enhance the electrochemical signal (Figs. 3 and 4). Increasing the current value can be attributed to the D_4_ concentration.

**Fig. 3:** Differential pulse voltammograms of **a** Ni(II) at Cit-Fe_3_O_4_-DMG-CPE; **b** Ni(II) and 300 ng/mL D_4_ at Cit-Fe_3_O_4_-DMG-CPE. Experimental conditions: pH 5, scan rate 100 mV s^−1^

**Fig. 4:** Schematic of Cit-Fe_3_O_4_-DMG carbon paste electrode

### Effect of supporting electrolyte, pH, deposing time& potential and scan rate

To achieve the high sensitivity, the effect of supporting electrolyte, pH, accumulation potential and scan rate on the electrode response were studied. To investigate the effect of electrolyte media and pH on the electrode response, various electrolytes such as sodium borate-boric acid, Britton-Robinson (B-R) and sodium acetate-acetic acid (HAc-NaAc) buffers were tested. The highest peak signal of D_4_ existed in the HAc-NaAc solution (0.05 M). While in sodium borate-boric acid, B-R solutions, weak peak signal were obtained. Consequently, in further experiments, HAc-NaAc (0.05 M) was chosen as the electrolyte. The pH of buffer solution has significant effect on the electrochemical signal of sensor. The influence of pH on the electrochemical response of Cit-Fe_3_O_4_-DMG-CPE electrode to D_4_ was studied. The results are presented in Fig. 5a. The results of this study show that by increasing the pH value up to 4.65, the peak signal of D_4_ increases. Then, the D_4_ electrochemical signal decreased with pH value up to 6.0. This result could be related to the deprotonation of HAc-NaAc buffer solution which promote the generation of H^+^, the concentration of D_4_ adsorbed on the Cit-Fe_3_O_4_-DMG-CPE surface would be less. Thus, the current signal of D_4_ would be increased with increase of pH till 4.65. With increase of pH from 4.65 to 6.0, the corresponding stripping signal was decreased due to the prevailing effect of D_4_ hydrolysis and formation of Ni(OH)_2_, Ni(OH)^+^, and Ni(OH)_3_^-^. Thus, pH 4.65 of HAc-NaAc buffer solution (0.05 M) was chosen in further experiments. In the electrochemical experiment, the accumulation potential is particularly vital for achieving good signals. In voltammetry, the deposition time has a significant impact on the electrochemical signals and sensitivity. The results of this study showed that the current signal D_4_ increased by increasing the accumulation time from 25 to 250 s (Fig. 5b). After 120 s, the signal intensity of D_4_ remained constant. Therefore the accumulation time of 120 s was selected for construction of the calibration curve and other experiments. The selection of 120 s as accumulation time was based on the development of a rapid method with a short real sample analysis time. In continue, the effect of accumulation potential on the electrode response was studied in the potential range of 0.0 to – 1.0 V (Fig. 5c). The results of this study show that by increasing the accumulation potential from 0.0 to – 1.0 V, the electrochemical signal is increasing till – 0.2 V and remains constant at more potential. At more negative accumulation potentials, reduction of D_4_ occurs, as indicated by decrease in the electrochemical signal of D_4_ measured during the scanning. Thus, – 0.2 V was adopted as the accumulate potential. Also, the effect of scan rate on the electrochemical signal of D_4_ showed that till 100 mVs^−1^, the response is increasing. It was shown that at scan rates from 0.1 to 100 mVs^−1^, the dependence of redox response upon the scan rate was linear which demonstrate an adsorption controlled process [24, 26]. The results of this study show that the cathodic and anodic peak current was increased with increasing the scan rate which indicates the oxidation and reduction process of D_4_ at Cit-Fe_3_O_4_-DMG-CPE electrode. So, it can be concluded that D_4_ was firstly absorbed on the electrode surface then the electrode reaction occurs.

**Fig. 5:** Effect of **a** pH; **b** deposition time; **c** deposition potential on differential pulse voltammograms of 250 ng/mL D_4_

### Calibration equation

Differential pulse voltammograms of different concentration of D_4_ at Cit-Fe_3_O_4_-DMG-CPE electrode in 0.05 M HAc-NaAc buffer at pH 4.65 are recorded (Fig. 6). It was shown that peak current values are linear at 50.0 to 340.0 ng/mL of D_4_ with regression equation of y(A) = 3E^−10^x(ng/mL)-2E^−08^ and correlation coefficient of R^2^ = 0.9834. The detection limit (3S_b_/m) of the electrode was calculated as 27.0 ng/mL. The results of this study reveal that the electrochemical voltammetry platform is sensitive to D_4_ determination.

**Fig. 6:** Calibration data. **a** Differential pulse voltammograms; **b** Calibration curve

### Stability, selectivity and repeatability

The reproducibility of Cit-Fe_3_O_4_-DMG-CPE electrode was excellent since the RSD (n = 10) was obtained as 3.8% which indicate the good repeatability of the electrode. The selectivity of electrode was evaluated by the determination of D_4_ in the presence of some potential interfering ions/molecules at optimized instrumental and operational conditions. Selectivity coefficient was defined as a concentration of the other ion/molecule that causes ± 5% relative error (RE) in the electrode response. The results of this study showed that most anions/cations and molecules Na^+^, Ca^2+^, Cu^2+^, Cu^+^, Fe^3+^, Fe^2+^, chlorate, iodate, bromate, chloride, bromide and thiosulfate don’t interfere with the system while Zn^2+^, EDTA, D_3_, D_5_ and D_6_, showed interference in D_4_ determination. However, the interference of EDTA and Zn^2+^ could be resolved by using them as potential masking agents for each others. As the results of interference study, major interference was found in the detection of low molecular weight (LMW) cyclic silicone families of D_4_ as D_3_, D_5_, and D_6_. Due to easy-to-use, inexpensive, non-GC methods are becoming increasingly popular for the determination of organic/organometallic substances including D_4_. To examine the stability of platform, in the 0.05 M of HAc-NaAc buffer 10 scan were made in the proposed potential range. The results show the voltammograms with clear background. Also, after 2 week storage of electrode in 0.05 M HAc-NaAc buffer, only 15% of electrochemical signals were decreased.

### Determination of D_4_ in urine and blood plasma

Blood and urine sample of workers of Ekbatan cement factory were collected. 1 mL of urine or blood plasma was transferred into a tube. After addition of 1 ml ethyl alcohol, each sample was vortexed. Then a certain amount of D_4_ was added to the samples and vortexed for 2 min. After addition of 2 mL hexane, the samples were re-vortexed for 2 min. It was transferred to the electrochemical cell and related voltammogram was recorded [25]. The results are presented in Tables 1 and 2.

**Table 1:** Determination of D_4_ in human blood plasma samples (n = 3)

Sample	Added (ng/mL)	Found (ng/mL)	Recovery (%)	Standard method^a^ (ng/mL)
Blood plasma	50.0	47.3	94.6	49.8
	100.0	92.0	92.0	96.3
	150.0	146.0	97.3	147.0
	200.0	193.2	96.6	197.4
	250.0	246.8	98.7	249.0

^a^GC-mass

**Table 2:** Determination of D_4_ in urine samples (n = 3)

Sample	Added (ng/mL)	Found (ng/mL)	Recovery (%)	Standard method^a^ (ng/mL)
Urine	50.0	46.9	93.8	48.4
	100.0	101.0	101.0	99.4
	150.0	148.0	98.6	150.3
	200.0	197.1	98.5	201.0
	250.0	244.3	97.7	246.9

^a^GC-mass

## Conclusions

In conclusion, the Cit-Fe_3_O_4_-DMG modified carbon paste electrode show superior detection capabilities as a result of enhances the electron transfer kinetics and surface area to volume ratio following the incorporation of Cit-Fe_3_O_4_ nanoparticles. The electrode has been successfully applied to the quantification of D_4_ in biological fluids.

## Data Availability

All data and materials could be available upon the request.

## Abbreviations

D_4_: Octamethylcyclotetrasiloxane
Cit-Fe_3_O_4_: Citrate stabilized Fe_3_O_4_
RSD: Relative standard deviation
LMW: low molecular weight
D_5_: decamethylcyclopentasiloxane
D_6_: Dodecamethylcyclohexa-siloxane
ICP: Inductively coupled plasma spectroscopy
HPLC: High performance liquid chromatography
GC: Gas chromatography
HAc-NaAc: Acetate-acetic acid
FTIR: Fourier-transform infrared spectroscopy
XRD: X-ray powder diffraction
VSM: Vibrating-sample magnetometer
SEM: Scanning electron microscope
B-R: Britton-Robinson

## References

[1] Mojsiewicz-Pieńkowska K, Jamrógiewicz M, Szymkowska K, Krenczkowska D (2016). Direct human contact with siloxanes (silicones)–safety or risk part 1. Characteristics of siloxanes (silicones). Front Pharmacol.

[2] CES–Silicones Europe. A Socio-Economic Study on Silicones. 2008, http://www.silicones.eu/uploads/Modules/Resources/ces-the-socio-economic-study_ brochure_v45.pdf 12

[3] Jebens AM, Kälin T, Kishi A, Liu S (2013). Chemical economics handbook, Denver.

[4] Frust K, The world silicone market: overview and forecasts, Proceeding of the International Silicone Conference, Fairlawn. 2014

[5] Schalau GK, Ulman KL, Silicone Excipients in Drug Development. Contra pharma. 2009. http://www.contractpharma.com/issues/2009- 06/view_ features/silicone-excipients-in-drug-development

[6] Rosendahl P, Hippler J, Schmitz OJ, Hoffmann O, Rusch P (2016). Cyclic volatile methylsiloxanes in human blood as markers for ruptured silicone gel-filled breast implants. Anal Bioanal Chem.

[7] Flassbeck D, Pfleiderer B, Klemens P (2003). Determination of siloxanes, silicon, and platinum in tissues of women with silicone gel-filled implants. Anal Bioanal Chem.

[8] Kala SV, Lykissa ED, Lebovitz RM (1997). Detection and characterization of poly(dimethylsiloxane)s in biological tissues by GC/AED and GC/MS. Anal Chem.

[9] Grumping R, Mikolajczak D, Hirner AV (1998). Determination of trimethylsilanol in the environment by LT-GC/ICP-OES and GC-MS. Fresenius J Anal Chem.

[10] Dudzina T, von Goetz N, Bogdal C, Biesterbos JWH, Hungerbühler K (2014). Concentrations of cyclic volatile methylsiloxanes in European cosmetics and personal care products: prerequisite for human and environmental exposure assessment. Environ Int.

[11] Horii Y, Kannan K (2008). Survey of organosilicone compounds, including cyclic and linear siloxanes, in personal-care and household products. Arch Environ Contam Toxicol.

[12] Wang RP, Moody R, Koniecki D, Zhu JP (2009). Low molecular weight cyclic volatile methylsiloxanes in cosmetic products sold in Canada: implication for dermal exposure. Environ Int.

[13] Xu L, Shi Y, Wang T, Dong Z, Su W, Cai Y (2012). Methyl siloxanes in environmental matrices around a siloxane production facility, and their distribution and elimination in plasma of exposed population. Environ Sci Technol.

[14] Xu L, Shi Y, Liu N, Cai Y (2015). Methyl siloxanes in environmental matrices and human plasma/fat from both general industries and residential areas in China. Sci Total Environ.

[15] Sánchez-Brunete C, Beatriz EM, Tadeo AJ (2010). Determination of cyclic and linear siloxanes in soil samples by ultrasonic-assisted extraction and gas chromatography-mass spectrometry. J Chromatog A.

[16] Parkinson GS (2016). Iron oxide surfaces. Surf Sci Rep.

[17] Heidarimoghadam R, Farmany A (2016). Rapid determination of furosemide in drug and blood plasma of wrestlers by a carboxyl-MWCNT sensor. Mater Sci Eng C.

[18] Heidarimoghadam R, Akhavan O, Ghaderi E, Hashemi E, Mortazavi SS, Farmany A (2016). Graphene oxide for rapid determination of testosterone in the presence of cetyltrimethylammonium bromide in urine and blood plasma of athletes. Mater Sci Eng C.

[19] Wei M, Zhao F, Feng S, Jin H (2019). A novel electrochemical aptasensor for fumonisin B_1_determination using DNA and exonuclease-I as signal amplification strategy. BMC Chem.

[20] Jin H, Wei M, Wang J (2013). Electrochemical DNA biosensor based on the BDD nanograss array electrode. Chem Central J.

[21] Farmany A, Shamsara M, Mahdavi H (2017). Enhanced electrochemical biosensing of buprenorphine opioid drug by highly stabilized magnetic nanocrystals. Sensor Actuat B.

[22] Badakhshan S, Ahmadzadeh S, Mohseni-Bandpei A, Aghasi M, Basiri A (2019). Potentiometric sensor for iron (III) quantitative determination: experimental and computational approaches. BMC Chem.

[23] Wahajuddin AS (2012). Superparamagnetic iron oxide nanoparticles: magnetic nanoplatforms as drug carriers. Inter J Nanomed.

[24] Mohammadi N, Najafi M, Adeh NB (2017). Highly defective mesoporous carbon ionic liquid paste electrode as sensitive voltammetric sensor for determination of chlorogenic acid in herbal extracts. Sensor Actuat B.

[25] Varaprath S, Seaton M, McNett D, Cao L, Plotzke KP (2000). Quantitative determination of octamethylcyclotetrasiloxane (D4) in extracts of biological matrices by gas chromatography-mass spectrometry. Intern J Environ Anal Chem.

[26] Abbasi S, Farmany A, Mortazavi SS (2010). Ultrasensitive simultaneous quantification of nanomolar level of Cd and Zn by cathodic adsorptive stripping voltammetry in some real samples. Electroanalysis.

